The article "Concurrent Associations between Physical Activity, Screen Time, and Sleep Duration with Childhood Obesity" was published in 2014. Journal: ISRN Obes.

# Concurrent Associations between Physical Activity, Screen Time, and Sleep Duration with Childhood Obesity

**DOI:** 10.1155/2014/204540

**Published:** 2014-03-09

**Authors:** Kelly R. Laurson, Joey A. Lee, Douglas A. Gentile, David A. Walsh, Joey C. Eisenmann

**Affiliations:** ^1^School of Kinesiology and Recreation, McCormick Hall, Illinois State University, Mailbox 5120, Normal, IL 61790, USA; ^2^Department of Psychology, Iowa State University, Ames, IA 50011, USA; ^3^Mind Positive Parenting, Minneapolis, MN 55406, USA; ^4^Division of Sports and Cardiovascular Nutrition, Department of Radiology, Michigan State University, East Lansing, MI 48823, USA

## Abstract

*Aim*. To examine the simultaneous influence of physical activity, screen time, and sleep duration recommendations on the odds of childhood obesity (including overweight). *Methods*. Physical activity was assessed via pedometer and screen time, and sleep duration were assessed via survey in a cross sectional sample of 674 children (aged 7–12 years) from two Midwestern communities in the fall of 2005. Participants were cross tabulated into four groups depending on how many recommendations were being met (0, 1, 2, or all 3). Linear and logistic regression were used to examine the influence of physical activity, screen time and sleep duration on obesity and interactions among the three variables. *Results*. Children achieving all three recommendations simultaneously (9.2% of total sample) were the least likely to be obese. Approximately 16% of boys and 9% of girls achieving all recommendations were overweight or obese compared to 53% of boys and 42.5% of girls not achieving any. *Conclusions*. The odds of obesity increased in a graded manner for each recommendation which was not met. Meeting all three recommendations appears to have a protective effect against obesity. Continued efforts are warranted to promote healthy lifestyle behaviors that include meeting physical activity, screen time, and sleep duration recommendations concurrently.

## 1. Introduction

Physical activity (PA), screen time (ST; i.e., television/video games), and sleep (SLP) are modifiable lifestyle risk factors for childhood obesity [1]. Many cross sectional and prospective studies have shown these variables to be independently associated with obesity [2–7]. As such, these variables are frequently studied in childhood obesity and, along with diet, are the specific focus of a recent Institute of Medicine statement on childhood obesity prevention [8].

In an attempt to promote general well-being and prevent or treat obesity, these risk factors are associated with clinical and public health recommendations. These recommendations include limiting ST to ≤2 hours per day, achieving ≥60 minutes of moderate to vigorous PA per day [9] (equivalent to 13,000 and 11,000 steps per day for boys and girls, resp.) [10], and sleeping 10-11 hours per night for children aged 5–12 years [11].

Independently, the effect of PA, ST, or SLP on obesity is well established. However, few studies have focused on these risk factors concurrently. We have previously found that children failing to meet both PA and ST recommendations were 3 to 4 times more likely to be obese than children meeting both [12]. Vioque et al. [13] showed that self-reported PA, ST, and SLP were predictive of obesity in Spanish adults (aged 15+ years) in a logistic model. Ortega et al. [14] found that 9-10 and 15-16 year old youth reporting more sleep also tended to report more PA and less ST. Based on these findings, interactions seem to exist between the three variables. However, further research is critical to determine to what extent this effect modification impacts obesity risk. Therefore, the purpose of this study was to examine the interactions between ST, SLP, and PA and determine their simultaneous influence on overweight and obesity using the aforementioned recommendations. This study can highlight the influence modifiable lifestyle risk factors may have on childhood obesity.

## 2. Methods

### 2.1. Participants

Participants in the study were from a childhood obesity intervention known as SWITCH [15]. SWITCH was a community, family, and school based intervention that took place in two school districts in Lakeville, Minnesota, and Cedar Rapids, Iowa. These two school districts were approached due to the requirements of funding agencies and all 10 elementary schools in the districts participated. Data for the current analysis are cross sectional in nature and were collected prior to randomization into treatment or control groups in the fall of 2005. Further details about SWITCH sampling and methods can be found elsewhere [15, 16]. Before study initiation, risks and procedures were explained verbally and in writing to all participants and their primary caregivers. Written consent and assent were obtained from the primary caregiver and child, respectively, prior to data collection. The study protocol was approved by the University of Minnesota's Human Subjects Review Board and is in accordance with the Declaration of Helsinki.

A total of 1,360 of 2,113 school children from two Midwestern communities were elected to participate in the intervention (64% response rate). Due to missing anthropometric measures, SLP, or ST data, or exclusion due to PA monitoring criteria (see below), the final analytic sample was 674 children. The overall demographics of the analytic sample are similar to the school districts from which the children were enrolled [15, 16].

### 2.2. Anthropometry

Stature was measured with a stadiometer (Seca Road Rod; Seca, Hamburg, Germany). Body mass was measured with a strain gauge scale (Lifesource MD; Lifesource, Milpitas, CA, USA). The growth charts of the Centers for Disease Control and Prevention [17] were used to determine individual BMI z-score and percentile. Children were classified as normal weight (BMI percentile <85), overweight (≥85th to <95th percentile), or obese (≥95th percentile).

### 2.3. Habitual Physical Activity

PA was assessed by pedometer (Digiwalker SW-2000), which is a suitable PA measuring device [18]. Accuracy of each pedometer was verified before data collection and participants were given instructions on wearing the pedometer. Participants recorded the number of steps taken each day over a 7-day period. Pedometer data were considered valid if the participants wore the monitor for ≥10 hours/day over ≥4 days (including at least one weekend day). Previous research supports this approach for characterizing PA [19]. Boys and girls were classified as meeting PA recommendations [10], if they averaged at least 13,000 and 11,000 steps per day, respectively.

### 2.4. Screen Time

Children reported how much time they spent watching television across the day, from waking to lunch, lunch to dinner, and dinner to bedtime. These questions were asked for a typical school day and for a typical weekend day. From this, average weekly television time was calculated. This procedure was repeated to assess video game playing. Weekly television and video game time were summed to provide a weekly estimation of total ST. This methodology of assessing ST has been used successfully in children before [20, 21]. Participants were grouped according to the American Academy of Pediatrics recommendation of no more than 2 hours per day of ST [9].

### 2.5. Sleep Duration

Average SLP was assessed by self-report and calculated in a method similar to ST. Children were asked what time they woke in the morning and what time they go to bed at night on a typical school day and then for a typical weekend day. SLP was characterized using the National Sleep Foundation recommendation of ≥10 hours of sleep per night [11].

### 2.6. Statistical Analysis

Gender and age specific z-scores were calculated for PA, ST, and SLP. These z-scores were summed for each participant to provide a combined risk factor z-score (after multiplying the ST z-score by −1). The combined z-score characterizes the child's overall placement in the sample for all three lifestyle variables. Higher z-scores indicate more PA, longer SLP duration, and less ST relative to the sample.

Descriptive statistics were calculated and means were compared between normal weight and obese children using independent* t*-tests. Frequency of meeting the PA, ST, and SLP guidelines were calculated for each recommendation and for combinations of those recommendations (i.e., meeting 0, 1, 2, or 3) along with the prevalence of overweight/obesity. Logistic regression was used to model the odds of meeting the PA, ST, or SLP recommendations using the other two recommendations (i.e., to determine whether children meeting the ST recommendation are more or less likely to meet the PA or SLP recommendations).

Partial correlations (adjusting for age, height, leg length, and ethnicity) were used to identify potential relationships among the risk factors and BMI percentile. Hierarchal linear regression was conducted using all lifestyle variables as continuous variables to quantify associations with BMI percentile (controlling for age, height, leg length, and ethnicity). The hierarchal models included all possible two- and three-way interactions. Standardized beta coefficients (Stan. *β*) were used to characterize each behavior's utility to predict BMI percentile (where 0.5 is the 50th percentile) even though different scales of measurement were used.

Logistic regression was used to determine what influence meeting the recommendations had on the odds of obesity. Models were stratified by gender and conducted with each risk factor independently and then in one full model including all three behavioral recommendations. Finally, we compared the odds of obesity between children meeting all, two, one, or none of the recommendations, combining boys and girls into one model and controlling for gender. Adequate fit and variance accounted for by the logistic models were determined using the Hosmer-Lemeshow test of goodness of fit and the Nagelkerke pseudo* r* ^2^. All data analyses were conducted using SPSS version 18 (Chicago, IL, USA).

## 3. Results

Descriptive statistics are provided in Table 1. One-third of the sample was overweight or obese, and these youth were taller (boys* t* = −3.49, *P* = 0.001; girls* t* = −5.26, *P* < 0.001), less active (boys* t* = 4.34, *P* < 0.001; girls* t* = 5.24, *P* < 0.001), engaged in more ST (boys* t* = −2.92, *P* = 0.004; girls* t* = −3.01, *P* = 0.001), and slept less (boys* t* = 3.07, *P* = 0.002; girls* t* = 2.69, *P* = 0.008) than normal weight children. Additionally, normal weight youth had a mean combined z-score in the upper half of the sample, compared to obese children with a mean combined z-score in the lower half (boys* t* = 5.75, *P* < 0.001; girls* t* = 6.26, *P* < 0.001). These differences were consistent for boys and girls excluding leg length, where normal weight girls had shorter legs (*t* = −2.55;  *P* = 0.011).

Table 2 shows the percentage of children that met the PA, ST, and SLP recommendations with the prevalence of overweight/obesity in each group. The bottom panel of Table 2 shows the percentage of children meeting all, two, one, or none of the recommendations. About 75% of youth met one or two of the three recommendations, with approximately 10% meeting all three and 15% meeting none. Of the 62 children meeting all three recommendations, 1 was obese (1.6%) and 6 were overweight (9.7%). In contrast, the prevalence of obesity in children not meeting any recommendations was approximately 26% with another 24% being overweight.

The correlation matrices examining the associations between BMI percentile and lifestyle variables are in Table 3. The strength of most correlations were low to moderate (e.g., *r* = 0.1–0.6). PA was significantly associated with BMI percentile in girls but not boys. Conversely, ST and SLP were significantly correlated to BMI percentile in boys, but not girls. The combined z-score showed the strongest correlation with BMI percentile (*r* = −0.23 in both boys and girls). Weak, inverse associations were found between SLP and PA and SLP and ST.

Results from logistic regression show that boys meeting the ST recommendation were 2.2 times more likely to also be meeting the SLP recommendation (1.2–3.8, *P* = 0.008). The results were similar for girls, where those meeting the ST recommendation were 2.0 times more likely to also be meeting the SLP recommendation (1.2–3.3, *P* = 0.007). Girls meeting the PA guidelines were 0.6 times less likely to also be meeting the SLP guidelines (0.4–0.9, *P* = 0.017) than girls not meeting the PA threshold.

For the hierarchal linear regression, all interactions (PA × ST, PA × SLP, ST × SLP, and PA × ST × SLP) were initially included but did not yield any significant predictors of BMI percentile. Therefore, none of the two- or three-way interactions were used in the final model. Results of the regression indicated that, when PA, ST, and SLP were entered within the same model, both PA and SLP were the strongest predictors of BMI percentile. ST had no significant association with BMI percentile in either the boys' or girls' model (both  *P* > 0.05). Specifically for boys, the standardized beta coefficients indicated that SLP (Stan. *β* = −0.172) was a better predictor of BMI percentile than PA (Stan. *β* = −0.119). However, the opposite was true for girls where the standardized *β* for SLP was −0.101 and the standardized *β* for PA was twice as large at −0.202.

Results of the logistic models predicting obesity are in Table 4. Generally, children failing to meet the PA and SLP recommendations were more likely to be obese than children that complied with the recommendations. However, when considered independently in the univariate models, the screen time recommendation alone was not a significant predictor of weight status in either boys or girls, and sleep duration was not a significant predictor for girls. However, all other logistic models had adequate fit when predicting weight status. When modeling all three recommendations concurrently, it appears that not meeting the PA recommendation is the strongest predictor of obesity. Girls and boys not meeting the PA recommendation were approximately 2.5 and 3 times more likely to be obese than children meeting the recommendations, respectively. Boys not getting the recommended amount of sleep were about 2.5 times more likely to be obese, but this association was not statistically significant for girls. In all, compared to children that met the three recommendations, those that failed one, two, and all three of the recommendations were approximately 2.5, 4.5, and 8.0 times more likely to be obese, respectively.

## 4. Discussion

The present study considered the concurrent influence of PA, ST, and SLP recommendations on childhood obesity. The main finding was that children meeting no risk factor recommendations were eight times more likely to be obese than those meeting all of the recommendations. The odds of obesity increased with each additional risk factor not being met. These variables appear to exert a synergistic effect on the odds of obesity when examined concurrently. For example, 50% of the children failing all three recommendations were overweight or obese, while only 11.3% of the children achieving all of the risk factors were overweight or obese. These results demonstrate the utility of these risk factor guidelines in respect to childhood obesity as well as quantify the impact of failing to meet multiple cutpoints simultaneously.

Few studies have examined the effects PA, ST, and SLP have on childhood obesity simultaneously. Martinez-Gomez et al. [22] found a positive association between the number of risk factors (PA, ST, SLP, and diet) and markers of adiposity in Spanish adolescents. Vioque et al. [13] found that obese Spanish adults spent more time watching TV and less time sleeping and were less active than nonobese individuals. They also found that television viewing time is a more important risk factor than PA in predicting obesity. In contrast, we found PA to be the most important risk factor for obesity. A potential reason for the disparity is that PA was assessed using different methodology. The strength of the association between physical activity and adiposity may depend on the method of measurement [23].

We found that children who spent more time sleeping spent less time being physically active. In contrast, Ortega et al. [14] found that youth who spent more time sleeping also tended to be more active. A potential reason for the inconsistency between studies might be due to differences in the methods that SLP and PA were quantified. Both studies assessed SLP via self-report, but Ortega et al. quantified sleep using categorical responses, while the current study had participants report sleep time as a continuous variable. Providing participants with categories to report sleep time restricts responses and may desensitize the impact of SLP. Also, Ortega et al. used weekday SLP, disregarding weekend sleep (though they did include weekend PA in the analysis). We calculated a weighted average of weekday and weekend SLP. Measuring weekend SLP may provide a more accurate estimate of overall SLP, especially when covarying for weekend PA. Since PA was objectively measured in the current study, it would make sense that children that wore the pedometer longer during the day would record more steps. Considering this, we used strict exclusion criteria (≥4 days with >10 hours/day of wear time) in hopes of decreasing any potential influence.

Unique aspects of the current study are the analytical design and specific attention to the interactions of PA, SLP, and ST. The study simultaneously examined three lifestyle risk factors for childhood obesity using established recommendations. As shown, the variables are correlated to some degree, making joint analyses of the variables critical to understanding their combined influence on childhood obesity. Further, we chose to focus on PA, SLP, and ST guidelines that practitioners use in the field. Therefore, the results provide practical and empirical evidence for clinicians, researchers, and policy makers.

Limitations of the study should be noted. Given the cross sectional design, it is not possible to determine whether not meeting current recommendations is the cause or outcome of obesity. Another limitation is the use of self-reporting for ST and SLP. Objective measurement was not feasible. However, both ST and SLP values reported here are comparable to national estimates [24, 25]. Finally, not all children in the school districts chose to participate in the intervention, which could lead to bias. However, when comparing the demographics of the analytic sample to those of the school districts the children were enrolled, there were no significant differences, indicating that the potential for bias is low.

## 5. Conclusion

Meeting the recommendations for PA, ST, and SLP appears to exert a robust protective effect from obesity. Compared to those meeting all three recommendations, children that failed to achieve any one, two, or all three were approximately 2.5, 4.5, and 8.0 times more likely to be obese, respectively. Only 1 of the 62 (1.6%) children meeting all three recommendations was obese. Continued efforts are warranted to promote healthy lifestyle behaviors that include meeting recommendations for physical activity, screen time, and sleep. Interventions should promote action for healthy levels of PA, ST, and SLP, instead of attempting to target them individually.

## Figures and Tables

**Table 1:** Descriptive statistics for boys and girls by weight status.

Variable	Boys		Girls	
	Normal weight	Overweight and obese	Normal weight	Overweight and obese
	(*n* = 206)	(*n* = 97)	(*n* = 245)	(*n* = 126)
Age (years)	9.7 (0.9)	9.6 (0.9)	9.6 (0.9)	9.7 (1.0)
Height (cm)	137.6 (7.1)	140.6 (7.1)*	136.5 (7.9)	141.1 (8.0)*
Leg length (cm)	65.4 (4.5)	66.3 (4.3)	65.2 (4.7)	66.5 (5.1)*
Weight (kg)	31.6 (4.6)	42.8 (8.6)*	30.8 (5.2)	45.2 (9.7)*
BMI (kg/m^2^)	16.6 (1.2)	21.5 (2.9)*	16.4 (1.5)	22.5 (3.0)*
Pedometer (steps/day)	13,382 (3,383)	11,647 (2,947)*	11,360 (2,461)	9,930 (2,550)*
Sleep duration (hours/day)	10.1 (1.0)	9.7 (1.0)*	10.3 (0.9)	10.1 (0.9)*
Screen time (hours/day)	4.2 (3.1)	5.4 (3.6)*	3.2 (2.3)	4.1 (2.9)*
Combined *z*-score	0.39 (1.7)	−0.83 (1.8)*	0.40 (1.6)	−0.78 (1.9)*

All values are mean SD.

*Overweight/obese significantly different from normal weight of same gender (*P* < 0.05).

Combined *z*-score = sum of age and gender specific *z*-scores from pedometer steps, sleep, and (inverse of) screen time.

**Table 2:** Percentage meeting physical activity, screen time, and sleep recommendations by overweight and obesity status.

Meeting recommendation	Boys (*n* = 303)			Girls (*n* = 371)			Full sample (*n* = 674)		
	Tot. (%)	Ov. (%)	Ob. (%)	Tot. (%)	Ov. (%)	Ob. (%)	Tot. (%)	Ov. (%)	Ob. (%)
Specific									
PA	42.2	13.3	7.0	45.0	17.4	8.4	43.8	15.6	7.8
ST	24.1	16.4	8.2	34.0	15.1	15.1	29.5	15.6	12.6
SLP	55.4	18.5	6.5	69.3	18.7	12.5	63.1	18.6	10.1
General									
Meet all	6.3	15.8	0.0	11.6	7.0	2.3	9.2	9.7	1.6
Meet 2 of 3	29.7	14.4	3.3	35.8	22.6	10.5	33.1	19.3	7.6
Meet 1 of 3	43.6	18.9	15.2	41.8	17.4	21.9	42.6	18.1	18.8
Meet none	20.5	30.6	22.3	10.8	12.5	30.0	15.1	23.5	25.5

Specific groups are not exclusive; youth may be represented in multiple groups.

Tot. (%) = percentage of total sample meeting the recommendation.

Ov. (%) = prevalence of overweight within group.

Ob. (%) = prevalence of obesity within group.

**Table 3:** Correlations between body mass index percentile and behavioral risk factors.

Variables	Girls (*n* = 371)				
	BMI percentile	Physical activity	Sleep duration	Screen time	Combined *z*-score
Boys (*n* = 303)					
BMI percentile	1	−0.22*	−0.10	0.10	−0.23*
Pedometer steps	−0.11	1	−0.13*	−0.04	0.51*
Sleep duration	−0.18*	−0.14*	1	−0.20*	0.60*
Screen time	0.12*	−0.06	−0.19*	1	−0.68*
Combined *z*-Score	−0.23*	0.51*	0.58*	−0.70*	1

*Statistically significant (*P* < 0.05).

Correlations adjusted for age, height, leg length, and ethnicity.

Combined *z*-score = sum of age and gender specific *z*-scores from pedometer steps, sleep, and (inverse of) screen time.

**Table 4:** Odds ratios for obesity using recommended guidelines for physical activity, screen time, and sleep.

Risk factor	Univariate model			Full model^a^		
	OR	95% CI	Nagelkerke *r* ^2^	OR	95% CI	Nagelkerke *r* ^2^
*Specific* ^ b^						
Boys failing to meet						
Physical activity	2.7	(1.6, 4.5)	0.065	3.1	(1.7, 5.5)	0.281
Screen time	1.5	(0.9, 2.9)	0.011	1.4	(0.7, 2.7)	—
Sleep	2.1	(1.3, 3.4)	0.039	2.4	(1.4, 4.3)	—
Girls failing to meet						
Physical activity	1.9	(1.3, 3.1)	0.034	2.5	(1.5, 4.2)	0.325
Screen time	1.3	(0.8, 2.1)	0.005	1.1	(0.7, 1.9)	—
Sleep	1.5	(0.9, 2.4)	0.011	1.6	(0.9, 2.8)	—
General						
Boys and girls						
Meeting all	Ref.	—	0.066	Ref.	—	0.291
Meeting 2 of 3	2.9	(1.3, 6.7)	—	2.6	(1.1, 6.5)	—
Meeting 1 of 3	4.6	(2.0, 10.5)	—	4.7	(1.9, 11.3)	—
Meeting none	7.6	(3.1, 18.1)	—	8.2	(3.2, 21.2)	—

^a^Adjusted specific models (boys *n* = 303; girls *n* = 371) controlling for age, height, leg length, ethnicity, and other risk factors (physical activity, sleep, and/or screen time). Adjusted general model (*n* = 674) controlling for age, height, leg length, ethnicity, and gender.

^b^Referent groups (OR = 1.0) are children meeting the specific recommendation.
